The article "Sufentanil Alleviates Sepsis-Induced Myocardial Injury and Stress Response in Rats through the ERK/GSK-3β Signaling Axis" was retracted in 2023. Reasons: signs of a paper mill; suspected computer-generated content; unreliable results or conclusions; concerns about the data.

# Sufentanil Alleviates Sepsis-Induced Myocardial Injury and Stress Response in Rats through the ERK/GSK-3*β* Signaling Axis

**DOI:** 10.1155/2022/9630716

**Published:** 2022-06-21

**Authors:** Hongcheng Zang, Gang Shao, Ying Lou

**Affiliations:** Department of Anesthesiology, The First People's Hospital, Fuyang, Hangzhou, Zhejiang 311400, China

## Abstract

**Objective:**

To explore the effect and possible mechanism of sufentanil on sepsis-induced myocardial injury and stress response in rats.

**Methods:**

The cecal ligation and puncture (CLP) method was utilized to establish the sepsis model of rats to explore the effect of sufentanil pretreatment with different concentrations on myocardial injury and oxidative stress in CLP rats. Echocardiogram was applied for detecting cardiac hemodynamic parameters in rats; hematoxylin and eosin (HE) staining as well as TUNEL staining was done for observing pathological changes of myocardial tissue and cardiomyocyte apoptosis in rats, respectively; biochemical testing and enzyme-linked immunosorbent assay (ELISA) were done for determining myocardial injury marker level in serum, oxidative stress substances in myocardial tissue, and neuroendocrine hormone level in serum of rats, respectively; finally, Western blot was performed for checking the expression level of ERK/GSK-3*β* signaling pathway-related proteins in myocardial tissue of rats.

**Results:**

A model of rat with sepsis-induced myocardial injury was constructed with the CLP method. Specifically, this rat model was characterized by obvious cardiac function and tissue damage, cardiomyocyte apoptosis, and oxidative stress response. Sufentanil pretreatment significantly improved cardiac function injury, alleviated pathological injury and oxidative stress response in myocardial tissue, and inhibited cardiomyocyte apoptosis. Specifically, after sufentanil pretreatment, left ventricular end-diastolic dimension (LVEDD) and left ventricular end-systolic dimension (LVESD) were downregulated, and left ventricular ejection fraction (LVEF) was upregulated; the level of *B*-type natriuretic peptide (BNP) of serum, creatine kinase isoenzyme (CK-MB), and troponin (cTnl) decreased; besides, malondialdehyde (MDA) level was declined, while activities of superoxide dismutase (SOD) and catalase (CAT) were increased. What is more, further mechanism exploration also revealed that sufentanil could reverse the activity of the sepsis-induced ERK/GSK-3*β* signaling pathway.

**Conclusion:**

Sufentanil has an obvious protective effect on myocardial injury and stress response in CLP rats, and this protective effect may be related to the activation of the ERK/GSK-3*β* signaling pathway.

## 1. Introduction

Sepsis is a systemic inflammatory response syndrome (SIRS) caused by an infection that occurs due to the invasion of various pathogenic microorganisms to the body [1]. Sepsis is a common complication for severe burns, ischemia-reperfusion (I/R), severe bleeding, and some surgical procedures, which can lead to septic shock and multiple organ dysfunction [2]. In fact, sepsis has already become one of the important causes of death in critically ill patients [2]. With the cases exceeding 30 million per year and 30% mortality, sepsis is undoubtedly one of the most urgent medical needs today [3]. Also, sepsis survivors have a higher rate of rehospitalization and are accompanied by a more severe condition [4]. Uncontrollable inflammatory response and refractory immunosuppression are considered as the major causes of poor prognosis in septic patients [5]. Myocardial tissue is a common target organ in sepsis, and myocardial tissue injury is the starting point for multiple organ dysfunction syndrome [6]. It is reported that cardiac structural damage occurs in the early stage of sepsis, and premature myocardial injury is associated with progressive deterioration of severe sepsis and high mortality [7]. Premature myocardial injury is a precursor of refractory shock. Moreover, this premature injury causes significantly increased mortality and is the key to resulting death in patients with sepsis [7]. Some other studies have shown that the mechanism of sepsis-induced myocardial injury is correlated with inflammation, oxidative stress, and myocardial apoptosis [8]. At present, the main treatment methods of sepsis include controlling inflammation and stress response and reducing myocardial injury.

Sufentanil is a synthetic opioid with advantages of strong lipid solubility, high attachment rate to human plasma proteins, good analgesic effect, hemodynamic stability maintenance, and is commonly used in patients undergoing cardiac surgery [9]. Studies reveal that sufentanil plays an important protective role in myocardial I/R injury [10–12]. Sufentanil has obvious protective effect on myocardial I/R injury in rats, and its mechanism may be related to activation of the ERK1/2 pathway and the inhibition of endoplasmic reticulum stress and oxidative stress [13, 14]. In addition, a study by Li et al. indicated a protective effect of sufentanil on skeletal muscle atrophy in septic patients [15]. Hu et al. revealed that sufentanil was able to reduce inflammation and oxidative stress in sepsis-induced acute lung injury [16]. ERK is a key extracellular-regulated protein kinase that achieves signal deliver from surface receptors to the nucleus, and can make cells function by modulating transcriptional activity [17]. ERK can be activated by phosphorylation, and p-ERK can promote Nrf2 phosphorylation. Specifically, p-Nrf2 enters the nucleus and bind to the corresponding promoters of target genes to promote downstream target gene expression, thereby exerting a protective effect on cellular function [17, 18]. GSK-3*β*, as a multifunctional serine/threonine kinase, plays an important role in myocardial injury. However, there are few reports on sufentanil in sepsis-induced myocardial injury. Based on the previous studies, we speculated that sufentanil may play a protective role in sepsis-induced myocardial injury. In order to verify above speculation, this study established a rat model of sepsis through the cecal ligation and puncture (CLP) method. Then the role of sufentanil in sepsis-induced myocardial injury and stress response in rats was assessed by echocardiogram, enzyme-linked immunosorbent assay (ELISA), biochemical testing, as well as HE staining. Additionally, we explored possible mechanism of action of sufentanil, providing a theoretical basis for its clinical application.

## 2. Materials and Methods

### 2.1. Experimental Animal

Beijing Vital River Laboratory Animal Technology Co., Ltd. provided 32 healthy SPF-grade SD male rats (Weight: 180–220* *g). The rats were adaptively housed at 20–23°C in a light/dark (12 h/12 h cycle) environment for 7 days, and all rats had free access to food and water. This study was approved by ethics committee of Guangdong Experimental Animal Center and conducted in accordance with the approved guidelines.

### 2.2. Establishment and Grouping of the Sepsis Rat Model

A rat model of CLP-induced sepsis was constructed according to the method in the study of Liu et al. [19]. Specifically, SD male rats were fasted but kept water supply for 24* *h before operation, then the rats were weighed and monitored general conditions. Subsequently, the rats were anesthetized through intraperitoneal injection of 50 mg/kg pentobarbital sodium followed by fixed shaving and routine abdominal disinfection. Then, a lower abdominal central incision (1.5 cm) was performed, and the cecum was exposed. After that, the cecum was ligated at 1 cm from the tip, and three perforations were carried out with an 18-gauge sterile needle in the central position of the distal cecal ligation. Finally, the cecum was placed back into the abdominal cavity, and then the abdominal incision was sutured layer by layer. Additionally, after surgery, 0.1 ml warm saline was injected subcutaneously to supplement fluid loss during surgery, and buprenorphine was injected subcutaneously to reduce postoperative pain. After operation, the rats showed delayed awakening, listlessness, hair erection, slow activity, reduced intake of food and water, slow response to the outside world, accelerated respiratory rate, and weak stool, suggesting that the sepsis model was successfully prepared.

Sufentanil was purchased from Yichang Humanwell Pharmaceutical Co., Ltd. Thirty-two SD rats were randomized into four groups (eight rats in each group). In the Sham group (*n* = 8), rats were injected with the same volume of normal saline as sufentanil in the tail vein. After 30 min, the rats were anesthetized, and the cecum was exposed without the CLP method. Other procedures were similar to the modeling group. In the CLP group (*n* = 8), rats were injected with the same amount of saline as sufentanil in the tail vein. After 30 min, the rats were anesthetized, and the CLP model was established by the CLP method. In the CLP + Suf 1 *μ*g/kg group (*n* = 8), sufentanil (1 *μ*g/kg) was injected into the tail vein of rats. After 30 min, the rats were anesthetized and the CLP model was constructed with the CLP method. In the CLP + Suf 3 *μ*g/kg group (*n* = 8), sufentanil (3 *μ*g/kg) was injected into the tail vein of rats. Then rats were anesthetized after 30 min. After that, the CLP method was utilized for the construction of the CLP model. Rats were anesthetized and subjected to echocardiogram 6 hours after CLP surgery, then the heart and blood samples were collected for index detection.

### 2.3. Determination for the Hemodynamic Indicators

Rats were anesthetized 6* *h after CLP surgery, then cardiac function measurements were performed in rats with a high-frequency ultrasound system and MS-250S probe (frequency: 13–24 MHz), respectively. Before surgery, the rats were weighed and then anesthetized with 2-3% isoflurane. After shaving the hair from the neck, chest, and abdomen with depilatory cream, the rats were supine, and fixed on a controlled heating pad to maintain their body temperature at 37°C. Subsequently, two-dimensional images of the left ventricle were obtained through a high-resolution probe. Then ten cardiac cycles were monitored under ultrasound guidance, and left ventricular end-diastolic dimension (LVEDD), left ventricular end-systolic dimension (LVESD), and left ventricular ejection fraction (LVEF) were also measured, and all electrocardiographic measurements were the mean of three cardiac cycles.

### 2.4. Examination of Biochemical Indicators

The plasma of rats was collected from the abdominal aorta and placed in an anticoagulant centrifuge tube. After centrifugation at 3500* *r/min for 15 min at 4°C, plasma supernatant was collected for subsequent trials. An automated biochemistry analyzer was applied for measuring the level of *B*-type natriuretic peptide (BNP), creatine kinase isoenzyme (CK-MB), and troponin (cTnl) in serum. Then rats were sacrificed, and the heart tissue was collected. Afterwards, malondialdehyde (MDA) content and activities of superoxide dismutase (SOD) and catalase (CAT) in myocardial tissue were measured according to the corresponding biochemical assay kit (Nanjing Jiancheng, China) instructions.

### 2.5. Pathological Observation of Myocardial Tissue

Rats were sacrificed, and the myocardial tissue was obtained, and then 4% paraformaldehyde solution was applied for fixation. Subsequently, the tissue was embedded, and cut into 5 *μ*m sections. After that, routine staining with hematoxylin and eosin (HE) was performed according to the instructions of HE staining kit (Beyotime Biotechnology, China). Finally, the pathological changes of myocardial tissue in each group were observed by a light microscope.

### 2.6. Apoptosis Examination

Cardiomyocyte apoptosis was assessed through terminal deoxynucleotidyl transferase dUTP nick-end labeling (TUNEL) assay. To be specific, myocardial tissue was fixed with 4% paraformaldehyde and then embedded and sliced. Subsequently, myocardial tissue sections were stained according to the TUNEL apoptosis detection kit (Solarbio, China) instructions. Specifically, phosphate-buffered saline (PBS) was adopted to wash the sections three times, then the nucleus was stained using DAPI solution (Solarbio) for 10 min. After that, the stain solution was rinsed with running water, and excessive water was absorbed with filter paper. One drop of fluorescent mounting solution was added, and then the sections were observed under a fluorescence microscope, and the images were collected; and apoptotic cells presented green fluorescence [20].

### 2.7. Detection for Adrenocorticotropic Hormone (ACTH) and Corticosterone (CORT)

The serum samples obtained in 1.4 were collected. Then the level of adrenocorticotropic hormone (ACTH) and corticosterone (CORT) in the serum of rats in each group was determined according to the corresponding ELISA kit (Nanjing Jiancheng, China) instruction.

### 2.8. Detection of Protein Expression Level

The myocardial tissue of rats was added into RIPA lysis solution (Solarbio, China) and then homogenized in a tissue homogenization instrument. Next, the tissue was lysed on ice for 30 min, then centrifuged at 10000 rpm for 20 min at 4°C. Subsequently, the supernatant of the protein was collected, and the concentration of total protein was checked with BCA kit (Beyotime Biotechnology, China). A total of 30 *μ*g total protein was added into loading buffer for denaturation treatment. Then sodium dodecyl sulfate polyacrylamide gel electrophoresis (SDS-PAGE) was conducted, and the protein was transferred onto polyvinylidene fluoride (PVDF) membrane (Merck Millipore, Germany). Further, the membrane was blocked in 5% skimmed milk for 2 h. After being washed by tris-buffered saline (TBST and 0.05% Tween 20) three times, the membrane was incubated with diluted primary antibodies (Proteintech, America) at 4°C overnight. Then the membrane was washed by TBST three times again, and diluted secondary antibodies (Proteintech, America) were added for another 1-h incubation at ambient temperature. TBST was utilized to wash the membrane for three times, and Western blot enhanced chemiluminescence (ECL) solution was dripped into the membrane. Finally, after being developed with gel imaging systems, the membrane was photographed. In addition, *β*-actin served as internal control and Image-pro plus software was adopted to analyze the relative protein expression.

### 2.9. Statistical Analysis

All results were presented as mean ± standard deviation (SD), and statistical analysis was performed with SPSS 22.0 software. *T*-test analysis was adopted for comparisons between two groups, and one-way analysis of variance for comparisons between multiple groups. *P* < 0.05 was considered as the judgment criterion of significant differences.

## 3. Results

### 3.1. Sufentanil Improves Cardiac Function and Alleviates Myocardial Injury in CLP Rats

The CLP method was adopted to construct the model of rats with sepsis for investigating the effect of sufentanil on sepsis. A series of echocardiographic and biochemical tests revealed that, compared with the Sham group (*n* = 8), the CLP group (*n* = 8) present a significant increase in LVEDD and LVESD (^*∗∗*^*P* < 0.01), while an obvious decrease in LVEF (^*∗∗*^*P* < 0.01), as well as a marked upregulation in the level of BNP, CK-MB, and cTnl in serum (^*∗∗*^*P* < 0.01) of rats. This result indicated the successful establishment of the CLP model of sepsis rats with impaired cardiac function. Additionally, compared with the CLP group (*n* = 8), rats with sufentanil treatment at different concentrations in the CLP + Suf 1 *μ*g/kg group (*n* = 8) and CLP + Suf 3 *μ*g/kg group (*n* = 8) showed a remarked decline in LVEDD and LVESD (^##^*P* < 0.01), a notable rise in LVEF (^##^*P* < 0.01), as well as a significant reduction in level of BNP (^#^*P* < 0.01), CK-MB and cTnl in rat serum (^##^*P* < 0.01) (Figures 1(a)–1(f)). Above results suggested sufentanil could effectively improve cardiac function and reduce myocardial injury in CLP rats.

### 3.2. Sufentanil Improves Myocardial Tissue Injury and Inhibits Myocardial Apoptosis in CLP Rats

The pathological changes of myocardial tissue in each group of rats were observed by HE staining. In the Sham group (*n* = 8), rats showed normal myocardial tissue structure, intact myocardial tissue morphology, as well as well-arranged myocardial fibers, and no obvious pathological changes were presented. In the CLP group (*n* = 8), rats presented diffuse interstitial edema, congestion, and hemorrhage, myocardial cell degeneration and necrosis, as well as myocardial fiber fragmentation, dissolution, and disarrangement, and accompanied by inflammatory cell infiltration. While pretreatment with sufentanil at 1 *μ*g/kg and 3 *μ*g/kg alleviated myocardial injury in rats, accompanied by a significant decrease in myocardial fiber and cardiomyocyte morphological abnormalities and inflammatory cell infiltration (Figure 2(a)). In addition, TUNEL staining revealed that apoptotic cells (TUNEL-positive) in the myocardial tissue of rats in the CLP group (*n* = 8) were significantly increased compared with those in the Sham group (*n* = 8). While TUNEL-positive cells in the myocardial tissue of rats in the CLP + Suf 1 *μ*g/kg group (*n* = 8) and CLP + Suf 3 *μ*g/kg group (*n* = 8) were markedly decreased and concentration-dependent (Figure 2(b)). All in all, sufentanil could ameliorate pathological injury of myocardial tissue and inhibit myocardial apoptosis in CLP rats.

### 3.3. Sufentanil Inhibits Oxidative Stress in Myocardial Tissue of CLP Rats

The effect of sufentanil on oxidative stress response in CLP rats was assessed by detecting the level of MDA (An oxidative stress product), SOD (A antioxidant enzyme), and CAT in myocardial tissue of rats in each group. The results indicated that compared with the Sham group (*n* = 8), the MDA content in myocardial tissue of rats in the CLP group (*n* = 8) was notably increased (^*∗∗*^*P* < 0.01), while the activities of SOD and CAT were markedly decreased (^*∗∗*^*P* < 0.01). Compared with the CLP group (*n* = 8), the MDA content in myocardial tissue of rats in the CLP + Suf 1 *μ*g/kg group (*n* = 8) and CLP + Suf 3 *μ*g/kg group (*n* = 8) significantly reduced (^##^*P* < 0.05), and the activities of SOD (CLP + Suf 1 *μ*g/kg group: ^#^*P*<0.05; CLP + Suf 3 *μ*g/kg group: ^##^*P* < 0.01) and CAT (CLP + Suf 1 *μ*g/kg group: ^##^*P* < 0.01; CLP + Suf 3 *μ*g/kg group: ^#^*P* < 0.05) were notably raised (Figures 3(a)–3(c)).

### 3.4. Sufentanil Declines the Level of Adrenocorticotropic Hormone (ACTH) and Corticosterone (CORT) in Plasma of CLP Rats

Patients with sepsis and septic shock typically present with increased plasma (free) cortisol (corticosterone in rodents; CORT) and suppressed plasma ACTH concentrations. In this paper, ELISA was conducted to determine the level of CORT and ACTH in plasma of CLP rats, and the results indicated that, compared with the Sham group (*n* = 8), ACTH and CORT level in plasma of rats in the CLP (*n* = 8) group was obviously raised (^*∗∗*^*P* < 0.01). Compared with the CLP group, the CLP + Suf 1 *μ*g/kg group (*n* = 8, ^##^*P* < 0.01) and CLP + Suf 3 *μ*g/kg group (*n* = 8, ^#^*P* < 0.05) showed a notably reduction in the level of ACTH and CORT in plasma of rats (Figures 4(a) and 4(b)). The above outcomes suggested that sufentanil could decrease the level of ACTH and CORT in plasma of CLP rats.

### 3.5. Sufentanil Regulates the ERK/GSK-3*β* Signaling Pathway in CLP Rats

It is reported that the ERK/GSK-3*β* signaling pathway played an important role in cardioprotection in a variety of diseases [21, 22]. While, it was unclear whether sufentanil could exert its function in cardiac injury of CLP rats. In this study, Western blot was applied to check the expression of ERK/GSK-3*β* signaling pathway-related proteins (p-ERK, ERK, p-GSK-3*β*, and GSK-3*β*) in myocardial tissues of rats in each group. As a result, compared with the Sham group (*n* = 8), myocardial tissues of rats in the CLP group (*n* = 8) presented much higher p-ERK level and p-ERK/ERK ratio (^*∗∗*^*P* < 0.01) and a lot lower p-GSK-3*β* level and p-GSK-3*β*/GSK-3*β* ratio (^*∗∗*^*P* < 0.01), while there were no significant differences between p-ERK and p-GSK-3*β* levels. Compared with the CLP group (*n* = 8), p-ERK and p-GSK-3*β* level and p-ERK/ERK and p-GSK-3*β*/GSK-3*β* ratios were notably increased (^*∗∗*^^##^*P* < 0.01), and the differences between ERK and GSK-3*β* expression levels were not statistically significant in the CLP + Suf 1 *μ*g/kg group(*n* = 8) and CLP + Suf 3 *μ*g/kg group (*n* = 8) (Figures 5(a) and 5(b)). Briefly speaking, sufentanil could activate the ERK/GSK-3*β* signaling pathway in CLP rats.

## 4. Discussion

As one of the commonly applied sepsis research models, the CLP rat model has high clinical relevance. As an important part of the circulatory system, the heart is one of the most vulnerable organs when sepsis occurs, and clinically, cardiac dysfunction is associated with increased mortality of sepsis [23, 24]. Also, animal experiments showed significantly attenuated cardiac function in septic rats [25]. In this study, the CLP rat model was constructed by the CLP method. Through HE staining and a series of biological indicators detection, we observed microstructural changes such as disarrangement, cell swelling, fiber fragmentation, and inflammatory infiltration in myocardial tissue of CLP rats, and normal hemodynamics, namely, cardiac dysfunction, was further presented. The above phenomena were basically consistent with the clinical findings of sepsis. While, after sufentanil pretreatment, myocardial injury and cardiac dysfunction were obvious improved, the level of BNP, CK-MB, and cTnl in serum was declined, and myocardial injury was relieved in CLP rats.

Sepsis-induced myocardial tissue mostly suffers from hypoxic-ischemic changes, and these changes cause apoptosis and necrosis of myocardial cells and then affect cardiac function [26]. In this paper, TUNEL assay exhibited a significant increase in TUNEL-positive apoptotic cells in myocardial tissue of rats in the CLP group; while after sufentanil intervention, the apoptotic cells in myocardial tissue declined. This outcome indicated the antiapoptotic effect of sufentanil on myocardial tissue in CLP rats. Some researches revealed a close relationship between sepsis and cardiomyocyte oxidative stress [27]. Sepsis declines the activity of oxygen-free radical scavengers in tissues, causing excessive oxygen-free radicals to be accumulated in tissues and can not be removed timely, and excessive oxygen-free radicals can induce lipid peroxidation, and then result in oxidative damage [28]. SOD and CAT, as antioxidant enzymes, are oxygen-free radical scavengers that present in the body [29]. MDA is the main product of lipid peroxidation [30], and a large number of oxygen free radicals in tissues can also activate apoptotic response and induce apoptosis [31]. In this research, SOD and CAT activities were decreased, and MDA level was increased in myocardial tissue of CLP rats, while sufentanil treatment could increase SOD and CAT activities and decline MDA level. This phenomenon indicated that sufentanil could improve oxidative stress caused by sepsis. Besides, sepsis increases myocardial apoptosis, then activates neuroendocrine system and results in massive secretion of stress hormones, thereby aggravating myocardial injury [32]. In this study, sufentanil decreased ACTH and CORT level in serum of CLP rats. The neuroendocrine system is involved in the immune regulation of sepsis through the release of hormones [33]. The corticotropin-releasing factor (CRH) is released from the hypothalamus to stimulate the anterior pituitary, and then releases ACTH into the circulation, and the circulating ACTH stimulates the adrenal glands Glucocorticoids are released [34]. Glucocorticoids in the blood regulate the further activation of the HPA axis through a feedback mechanism mediated by the glucocorticoid receptor (GR) in the brain. When the HPA axis is activated during sepsis, the adrenal cortex releases CORT to induce anti-inflammatory effects of immune cells (including macrophages, monocytes, and neutrophils) [34]. It is suggested that sufentanil could inhibit neuroendocrine activation, reduce stress hormone secretion, and then play a role in protecting cardiac function.

It has been reported that activation of GSK3*β* by phosphorylation can obviously reduce oxidative stress response, inflammatory response, and cardiomyocyte apoptosis in the myocardium, thereby reducing myocardial injury [35]. In addition, Nudelman et al. disclosed that AN-7 played a protective role in hypoxia-induced myocardial injury by inducing the phosphorylation of ERK as well as downstream GSK-3*β* [36]. Through detecting ERK/GSK-3*β* signaling pathway-related protein level, this study revealed that the level of p-ERK and p-GSK-3*β* and the ratios of p-ERK/ERK and p-GSK-3*β*/GSK-3*β* in the myocardial tissue of CLP rats increased markedly after sufentanil treatment. The above finding suggested that sufentanil may relieve sepsis-induced myocardial injury and stress response in rats by activating the ERK/GSK-3*β* signaling pathway. We only determined the effect of sufentanil on the ERK/GSK-3*β* signaling pathway, and it is still unclear for other molecular mechanisms of sufentanil. For instance, it was reported that sufentanil increases the growth rate in H9C2 cells through activation of ERK1/2 pathway [13]. Sufentanil appears to be beneficial in patients with worsening ischemic heart disease. Wu et al. reported that sufentanil pretreatment could prevent myocardial I/R injury via the miR-125a/DRAM2 axis [37]. In I/R rats, sufentanil alleviates myocardial injury and plays a protective role by inhibiting oxidative stress, inflammatory response, and endoplasmic reticulum stress [14]. Therefore, further exploration to sufentanil is required. In conclusion, our study revealed that sufentanil played a significant protective role in sepsis-induced myocardial injury and oxidative stress, but whether it could be applied in the clinical treatment of sepsis needs further clinical trial evaluation.

## 5. Conclusion

To sum up, sufentanil can relieve cardiac function injury, myocardial tissue injury and stress response, and inhibit cardiomyocyte apoptosis in CLP rats. Additionally, mechanism of action of sufentanil may be achieved by activating the ERK/GSK-3*β* signaling pathway, and its specific mechanism requires further investigation.

## Figures and Tables

**Figure 1:** Sufentanil can effectively improve cardiac function and relieve myocardial injury in CLP rats. (a)–(c) Echocardiographic assessment of cardiac function-related parameters in each group of rats, including left ventricular end-diastolic dimension (LVEDD (a)), left ventricular end-systolic dimension (LVESD (b)), and left ventricular ejection fraction (LVEF (c)). (d)–(f) Biochemical testing applied to determine the level of myocardial cell injury-indicators BNP (d), CK-MB (e), and cTnl (f) in serum of rats in each group. ^*∗∗*^*P* < 0.01 vs. the Sham group, ^#^*P* < 0.05 and ^##^*P* < 0.01 vs. the CLP group.

**Figure 2:** Sufentanil ameliorates cardiac tissue injury and inhibits myocardial apoptosis in CLP rats. (a) HE staining performed to observe the pathological injury of myocardial tissue in each group; (b) the level of apoptosis in the myocardial tissue of rats in each group assessed by TUNEL staining.

**Figure 3:** Sufentanil suppresses oxidative stress in myocardial tissue of CLP rats. (a)–(c) Biochemical testing for the content of MDA (a) and the activities of SOD (b) and CAT (c) in myocardial tissue of rats in each group. ^*∗∗*^*P* < 0.01 vs. the Sham group, ^#^*P* < 0.05 and ^##^*P* < 0.01 vs. the CLP group.

**Figure 4:** Sufentanil decreases the level of ACTH and CORT in plasma of CLP rats. (a)-(b) The level of ACTH (a) and CORT (b) in plasma of CLP rats checked by ELISA. ^*∗∗*^*P* < 0.01 vs. the Sham group, ^#^*P* < 0.05 and ^##^*P* < 0.01 vs. the CLP group.

**Figure 5:** Sufentanil regulates the ERK/GSK-3*β* signaling pathway in CLP rats. (a) Western blot for detecting the level of ERK/GSK-3*β* signaling pathway-related proteins (p-ERK, ERK, p-GSK-3*β*, and GSK-3*β*) in myocardial tissues of rats in each group; (b) image *J* software utilized to analyze the ratios of p-ERK/ERK and p-GSK-3*β*/GSK-3*β* in myocardial tissues of rats in each group, ^*∗∗*^*P* < 0.01 vs. the Sham group, ^#^*P* < 0.01 vs. the CLP group.

## Data Availability

The data used to support the findings of this study are available from the corresponding author upon request.
